The article "Menopausal Symptoms and Sleep Quality in Women Aged 40–65 Years" was retracted in 2023. Reasons: unreliable results or conclusions; lack of ethics approval or compliance; concerns about the data; concerns about the results or conclusions.

# Menopausal Symptoms and Sleep Quality in Women Aged 40–65 Years

**DOI:** 10.1155/2022/2560053

**Published:** 2022-08-09

**Authors:** Zicheng Song, Rongzhen Jiang, Changbin Li, Feng Jin, Minfang Tao

**Affiliations:** Department of Obstetrics and Gynecology, Shanghai Jiao Tong University Affiliated Sixth People's Hospital, Shanghai 200233, China

## Abstract

The study examined the relationship between menopausal symptoms and sleep disturbances and the related influencing factors. *Methods*. We recruited women aged 40-65 years who attended the menopause clinic at Shanghai Jiao Tong University's Sixth People's Hospital from February 2011 to November 2019. The Menopause Rating Scale (MRS) was used to collect women's menopausal symptoms, and the Pittsburgh Sleep Quality Index (PSQI) was used to evaluate the subjects' sleep condition. We used logistic regression models to identify the relationship between menopausal symptoms and sleep quality. *Results*. A total of 1341 participants were recruited in this study. The most frequent three symptoms assessed by MRS were fatigue (72.9%), sleep disturbance (67%), and hot flashes with night sweats (65%). Participants' age was significantly associated with the severity of menopausal syndrome (*P* < 0.01). According to the PSQI sleep evaluation, 66.9 percent of participants had sleep disturbances (PSQI > 5). Logistic regression analysis revealed that women with mild, moderate, or severe menopausal syndrome had a 3-, 7-, and 17-fold increased chance of having sleep disturbances compared to women without menopausal syndrome. *Conclusion*. Women aged 40–65 years were found to have a significantly higher risk of menopausal syndrome and sleep disturbances.

## 1. Introduction

Menopausal syndrome and sleep disorders are extremely common in (peri)menopausal women very often. Menopausal syndrome has a general prevalence of 50-82%, varying according to race and region [1, 2]. The most predominant symptom of menopausal syndrome is hot flush. Study indicates up to 80 percent of women experience the vasomotor syndrome [3]. Vasomotor symptoms (VMS) at night can cause major sleep disruptions in a number of women [4, 5]. Studies indicate that the vasomotor syndrome is associated with 27-69 percent of night awakening [6, 7]. Even though vasomotor syndrome is highly associated with sleep disturbance in menopause, there are several other sleep-disrupting factors that detriment sleep qualities [8]. Some menopausal women suffer from sleep problems even when they are not experiencing hot flashes. Sleep disorders are prevalent in perimenopausal women at a rate of 32-46% [9, 10]. Additionally, several studies have discovered an increasing prevalence of sleep problems with advancing age [11, 12]. Not only do sleep disorders impair the life quality of (peri)menopausal women but they also have a greater impact on women's cardiovascular systems. It is an independent risk factor for atherosclerosis in menopausal women [13] and can lead to a significant increase in cardiovascular disease [14].

The article "Menopausal Symptoms and Sleep Quality in Women Aged 40–65 Years" was retracted in 2023. Reasons: unreliable results or conclusions; lack of ethics approval or compliance; concerns about the data; concerns about the results or conclusions.

The prevalence of menopausal sleep problems varies by region [15]. Europe has the highest incidence at 74%, North America has a prevalence of 36-50%, Latin America has a prevalence of 45-69%, and Asia has a prevalence of 22-63% [16].

## 2. Methods

### 2.1. Study Subjects

The subjects of this study were women who visited the menopausal clinic at Shanghai Jiao Tong University's Sixth People's Hospital and willingly completed a questionnaire survey between 2 January 2011 and 11 January 2019. The following criteria were used to determine inclusion: (1) age 40–65 years, (2) Shanghai household registration or residency in Shanghai for a period of at least five years, (3) no prior psychopsychiatric disorders, (4) no prior sleep disorders, and (5) voluntary participation and signed informed consent form. Exclusion criteria include the following: (1) individuals who have received menopausal hormone therapy within the last six months, (2) individuals who have received traditional Chinese medicine or other treatments for alleviating menopause-related symptoms within the last six months, and (3) individuals who have serious organic diseases. During the investigation period, a total of 1341 study subjects were enrolled. The study was approved by the Ethics Committee of Shanghai Jiao Tong University's Sixth People's Hospital.

### 2.2. Data Collection

From February 2011 to November 2019, our study's leading researchers performed a weekly clinic for menopausal symptoms at Shanghai Sixth's People Hospital. Once patients met the inclusion criteria and provided informed consent, three to four researchers with professional training would collect participants' demographic information, inquire about their past medical history, and administer the standardized screening tools, such as the Menopause Rating Scale (MRS) and Pittsburgh Sleep Quality Index (PSQI). In addition, their prescriptions for symptom treatment would be recorded for future consultation.

#### 2.2.1. Demographic Data

The study subjects' age, marital status, employment status, per capita monthly income, education level, and body mass index (BMI) were determined using a self-administered questionnaire. According to the Guidelines for the Prevention and Control of Overweight and Obesity in Chinese Adults, BMI < 18.5 kg/m^2^ was considered as underweight; BMI 18.5~23.9 kg/m^2^ was considered normal body mass; BMI > 24 kg/m^2^ was considered obese [17].

The article "Menopausal Symptoms and Sleep Quality in Women Aged 40–65 Years" was retracted in 2023. Reasons: unreliable results or conclusions; lack of ethics approval or compliance; concerns about the data; concerns about the results or conclusions.

#### 2.2.2. Standard Screening Tools

Menopausal symptoms were assessed using the Menopause Rating Scale (MRS), with an overall reliability coefficient ranging from 0.6 to 0.9 across countries [18]. Menopausal symptoms and their severity were assessed using the Menopause Rating Scale (MRS). The scale consisted of eleven questions, each of which was assigned a score of 0, 1, 2, 3, and 4 to represent normal, mild, moderate, severe, or extremely severe symptoms, for a total score of 44. Heinemann defined the severity scale as follows: 0~4 was considered normal, 5~8 was considered mild, 9~15 was considered moderate, and over 16 was considered extremely severe [18].

PSQI was used to assess the participants' sleeping status, with an overall reliability coefficient (Cronbach's *a*) of 0.83. A total PSQI score of >5 is frequently regarded as threshold for diagnosing sleep disorders [19]. In a Shanghai study, the diagnostic criteria were 8 [12]. In this study, we defined PSQI score over 5 as insomnia. The PSQI scale consisted of seven major categories, each of which contained 19 distinct questions. Each category assigned a point value to the severity of sleep disorders ranging from 0 to 3, with a maximum of 21. In addition, the prevalence of sleep disorders in women aged 40-65 years in Shanghai is evaluated to explore the relationship between menopausal syndrome and sleep quality, which help us generate appropriate preventive and management measures.

#### 2.2.3. Data Analysis

The database was created using Excel 2016, and statistical analysis was performed using SPSS 25.0 software. Frequency and percentage were used to describe categorical data, while mean ± standard deviation was calculated to describe quantitative data descriptively. The categorical data was compared using chi-square test to determine differences in menopausal symptoms and sleep quality between subjects with varying characteristics. Binary logistic regression models were performed to explore factors associated with the sleep quality, with *P* < 0.05 considered statistically significant.

## 3. Results

### 3.1. Demographic Characteristics of the Study Subjects

A total of 1341 study subjects were recruited, aged 51.43 ± 5.28 years, with 13.8% (185/1341) in the 40-44 age group, 28.3% (380/1341) in the 45-49 age group, 36.8% (494/1341) in the 50-54 age group, and 21% (282/1431) in the 55-65 age group. BMI was 23.81 ± 62.29 in average, with 65.2% of the population having a normal BMI, 6.6% being underweight, and 22.1% being overweight. 58.5% of study subjects were employed. The greatest percentage of household per capita monthly income was RMB 3000-4999 (31.45%). In terms of educational attainment, 48.5% had completed middle school or less, followed by high school (32.5%). See Table 1.

The article "Menopausal Symptoms and Sleep Quality in Women Aged 40–65 Years" was retracted in 2023. Reasons: unreliable results or conclusions; lack of ethics approval or compliance; concerns about the data; concerns about the results or conclusions.

#### 3.1.1. The Prevalence and Factors for Menopausal Symptoms

Menopausal syndrome was prevalent in 76.1% (1020/1341) of the study individuals, with prevalence rates of 24.8% (333/1341), 35.0% (469/1341), and 16.3% (219/1341) for mild, moderate, and severe symptoms, respectively. 73% (1289/1720) of participants experienced physical or mental exhaustion. 67% (1162/1720) reported experiencing sleep difficulties. Hot flashes were prevalent in 65% (1130/1720) of the people. Other common symptoms were followed by joint/muscle discomfort (61%, 1070/1720), irritation (48%, 842/1720), cardiac discomfort (48%, 896/1720), depression (46%, 811/1720), anxiety or panic (46%, 810/1720), and genitourinary tract symptoms (43%, 761/1720). In less than 35% of cases, problems such as decreased libido and trouble peeing occurred. For further information, see Figure 1.

#### 3.1.2. Risk Factors for the Severity of Menopausal Syndrome

It was discovered that the proportion of women with normal or mild menopausal syndrome was higher in the younger age group, while the proportion of women with moderate or severe menopausal syndrome was higher in the older age group, and their differences were statistically significant (*P* < 0.001). BMI was not statistically associated with the severity of menopausal syndrome. See Table 2.

### 3.2. Menopausal Sleep Quality and Its Association with Age, BMI, and MRS

966 individuals (69.6%) experienced sleep problems, with 54.1% (100/154) in the 40-44 age group, 66.8% (254/380) in the 45-49 age group, 75.3% (372/494) in the 50-54 age group, and 76.2% (215/282) in the 55-65 age group. Sleep disturbances occurred in more than 75% of groups above the age of 50. The difference in sleep problem prevalence across age groups was statistically significant (*P* < 0.001). The difference of sleep disturbances between levels of BMI was not statistically significant. Additionally, a strong positive correlation between menopausal symptoms and sleep quality was identified. Participants with little or moderate menopausal symptoms were more likely to report primarily normal or mildly impaired sleep quality, whereas participants with severe menopausal symptoms reported a significantly higher risk of sleep problems (*X* = 211.9, *P* < 0.001). Observe Table 3.

### 3.3. Sleep-Related Risk Factors

The multivariate logistic regression model was employed to identify the association between menopausal syndrome and sleep disorders by controlling potential confounders. Results showed that women with mild, moderate, or severe MRS were almost threefold (OR 2.76, 95% CI in 1.96~3.88), sevenfold (OR 6.61, 95% CI 4.64~9.44), and seventeenfold (OR 6.61, 95% CI 4.64~9.44) more likely having sleep disorders, respectively. There was no statistically significant difference between women's age, BMI, marital status, employment status, education level, family income, dysmenorrhea, menopausal status, or sleep disruption in the research individuals. See Table 4.

The article "Menopausal Symptoms and Sleep Quality in Women Aged 40–65 Years" was retracted in 2023. Reasons: unreliable results or conclusions; lack of ethics approval or compliance; concerns about the data; concerns about the results or conclusions.

## 4. Discussion

### 4.1. Epidemiology of Menopausal Symptoms

Menopausal syndrome has long had an adverse effect on women's quality of life. In the 1960s, developed nations launched interventions for menopause-related health issues [20]. China, on the other hand, lagged far behind. Nowadays, menopausal population health management has become increasingly important and crucial due to the current rapid growth in aging, along with a growing population. A substantial number of studies on the clinical symptoms of menopause have been undertaken domestically and internationally. However, findings differ slightly between publications due to difference of study methods, sample sizes, and participants. In our study, 79% of women between the ages of 40 and 65 years suffer from menopausal syndrome. This finding is consistent with the preponderance of women along the southeast region [21, 22], but is notably contrary to the findings reported for the northern area [23]. The primary causes for the difference might be due to changes in sample technique, living environment, and features among others [21].

Locally tailored preventive and consultation programs should be developed in each location, taking into account the prevalence and severity of menopausal syndrome. In our study, sleep disturbance was the second most frequent clinical symptom among women aged 40 to 65, following physical and mental fatigue (72.9 percent). The major clinical manifestations discussed in current textbooks in China are based on researches conducted in Europe and the United States, where the primary symptom in menopausal women in the United States was hot flashes and night sweats (87%) [24], with a significantly higher prevalence of diastolic symptoms in African-Americans and Hispanics than in Asians [25], and sleep disturbances at 32-48% [10]. As a result, menopausal syndrome care in China requires a comprehensive strategy built on relevant epidemiological and clinical studies.

### 4.2. Association between Menopause and Sleep Quality

This study establishes a link between sleep quality and the severity of sleep disturbances and menopausal syndrome. Sleep disturbances are 2.75, 6.61, and 16.83 times more likely to occur in individuals with varying degrees of menopausal syndrome than in women who do not have it. Menopausal sleep quality is unrelated to menopause status but is connected with the severity of menopausal symptoms [26], which is consistent with our findings. Insomnia is more prevalent in menopausal women [27], and it is commonly connected with anxiety and sadness [28]. This may help to explain why, in contrast to hot flashes and night sweats, hormone treatment alone is unable to completely resolve sleep difficulties [28], since the etiology and presentation of sleep disorders are more complicated.

The article "Menopausal Symptoms and Sleep Quality in Women Aged 40–65 Years" was retracted in 2023. Reasons: unreliable results or conclusions; lack of ethics approval or compliance; concerns about the data; concerns about the results or conclusions.

Menopausal symptoms and sleep disturbances have a reciprocal influence [4, 5]. During menopausal symptoms, sleep disturbances are frequently cooccurring with other mental diseases such as anxiety and depression [28]. Sleep-related symptoms such as difficulties in beginning or sustaining sleep were worsened, resulting in impaired daytime function [29]. By comparing objective measures such as the sleep tester to patients with insomnia, it has been demonstrated that individuals with insomnia tend to overestimate their time spent asleep and underestimate their overall sleep time. This demonstrates that the patient's attitude towards their sleep issues has a significant role in the assessment, diagnosis, and treatment of insomnia [30].

As a result, we should pay more attention to sleep disturbances among Shanghai's menopausal women. Together with menopausal medication, appropriate psychotherapy to alter patients' misperceptions may be effective in alleviating the severity of the menopausal syndrome. More clinical studies are required to evaluate the feasibility. Menopausal symptoms often persist years (7.4 years on average) and vary according to ethnic group and regions [31].

### 4.3. Other Factors Affecting Sleep

Concerning the etiological therapy, further exploration of the processes by which menopausal syndrome and sleep quality interact is required. For the time being, it appears as though long-term sleep issues are inextricably linked to physiological activity [32]. Additionally, insomniacs have decreased hypothalamus activity and caused a shrinkage of the hippocampus [33, 34]. However, it is uncertain if this holds true for menopausal women.

The results of this study reveal that age, BMI, and education level of menopausal women have no influence on sleep quality. It is worth mentioning that age has a positive link with the severity of Menopause Rating Scale but not with sleep disorders. In comparison, the finding indicates that age is a significant predictor of insomnia and predisposes individuals to acquire sleep disorders [27]. The disparity is partly explained by a small sample size, which renders age statistically insignificant. Therefore, we are unable to apply the STRAW categorization for diagnosis of menopausal women's sleep problems since it does not identify the severity of sleep disorders [35], hence precluding its usage. Additionally, we advocate for increased sleep research with the goal of quantifying and analyzing the repercussions of sleep disturbances.

The article "Menopausal Symptoms and Sleep Quality in Women Aged 40–65 Years" was retracted in 2023. Reasons: unreliable results or conclusions; lack of ethics approval or compliance; concerns about the data; concerns about the results or conclusions.

### 4.4. Limitations

In this paper, the participants were only from single hospital outpatients. A small number of subjects were not cooperative for interviews, so there was some response bias. In addition, the study did not control the homogeneity of hormone levels, which may have biased the results.

## 5. Conclusion

The results of this study indicate that women with menopausal syndrome in Shanghai had a high prevalence of sleep disturbances. Menopausal symptoms are strongly correlated with the degree of sleep disorders. Menopausal syndrome palliation may alleviate the severity of sleep disorders in women.

## Figures and Tables

**Figure 1:** Distribution of perimenopausal symptoms in study subjects (%).

**Table 1:** Demographic characteristics of study population.

Object characteristics	Number of people	%
Age (years)		
40~44	185	13.8
45~49	380	28.3
50~54	494	36.8
55~65	282	21.0
Marriage		
Married	1307	97.5
Other	34	2.5
Working status		
Retirement	490	36.5
Occupation	785	58.5
Other	66	4.9
Monthly per capita household income (RMB)		
2999 or below	272	20.3
3000-4999	421	31.4
5000-9999	345	25.7
10000 or above	303	22.6
BMI (kg/m^2^)		
<18.5	89	6.6
18.50~23.9	875	65.2
≥24	296	22.1
Education background		
Primary and illiterate	188	14.0
Middle school	651	48.5
High school	436	32.5
University and above	66	4.9

**Table 2:** Characteristics and significance of menopausal syndrome.

Object characteristics	Severity of menopausal syndrome				
	*N* ^#^	Normal	Mild	Moderate	Severe
Age (years)^∗∗∗^					
40~44	180	80 (44.4%)	45 (25.0%)	35 (19.4%)	20 (11.1%)
45~49	376	101 (26.9%)	111 (29.5%)	120 (31.9%)	44 (11.7%)
50~54	485	88 (18.1%)	102 (21.0%)	201 (41.4%)	94 (19.4%)
55~65	279	47 (16.8%)	69 (24.7%)	106 (38.0%)	57 (20.4%)
BMI					
<18.5	87	20 (23.0%)	20 (23.0%)	35 (40.2%)	12 (13.8%)
18.5~24.0	864	224 (25.9%)	213 (24.7%)	288 (33.3%)	139 (16.1%)
≥24	290	55 (19.0%)	67 (23.1%)	117 (40.3%)	51 (17.6%)

^∗∗∗^ *P* < 0.001.

**Table 3:** Stratified analysis of sleep quality severity.

Object characteristics	PSQI			
	0-5	>5	*X* ^2^	*P*
Age			36.152	<0.001
40~44	85 (45.9%)	100 (54.1%)		
45~49	126 (33.2%)	254 (66.8%)		
50~54	122 (24.7%)	372 (75.3%)		
55~65	67 (23.8%)	215 (76.2%)		
BMI			4.346	0.114
18.50	23 (25.8%)	66 (74.2%)		
18.50~24.00	276 (31.5%)	599 (68.5%)		
≥24	76 (25.7%)	220 (74.3%)		
MRS			219.467	<0.001
Normal	185 (58.5%)	131 (41.5%)		
Mild	113 (34.6%)	214 (65.4%)		
Moderate	78 (16.9%)	384 (83.1%)		
Severe	15 (7.0%)	200 (93.0%)		

The article "Menopausal Symptoms and Sleep Quality in Women Aged 40–65 Years" was retracted in 2023. Reasons: unreliable results or conclusions; lack of ethics approval or compliance; concerns about the data; concerns about the results or conclusions.

**Table 4:** Multiple regression analysis of factors influencing sleep disorders.

	Adjusted OR	OR 95% confidence interval	
		Lower limit	Upper limit
MRS			
Normal	1		
Mild	2.755	1.956	3.881
Moderate	6.614	4.635	9.438
Severe	16.827	9.381	30.183
Age (years)			
40~44	1		
45~49	1.313	0.864	1.997
50~54	1.493	0.948	2.353
55~65	1.368	0.796	2.351
BMI			
18.5~24.0	1		
<18.5	1.382	0.788	2.422
≥24	1.097	0.783	1.535
Marital status			
Married	1		
Other	1.116	0.458	2.720
Status of employment			
Retirement	1		
Incumbency	1.146	0.783	1.678
Missing	0.762	0.374	1.552
Education level			
Middle school	1		
University	0.539	0.330	0.879
High school	0.707	0.438	1.141
Primary school	0.748	0.350	1.599
Household income per capita			
≥10000	1		
≤2999	0.972	0.595	1.587
3000~4999	0.999	0.671	1.487
5000~9999	0.952	0.626	1.448
Menopausal status			
Premenopause	1		
Menopause	1.265	0.822	1.946
Missing	1.216	0.345	4.288

## Data Availability

The data that support the findings of this study are available from the corresponding author upon reasonable request.
